# Feasibility Analysis of Mutual Benefit Cooperation between Environment-Embedded Art Design Education and Local SMEs Development Based on Improved Grey Analysis

**DOI:** 10.1155/2022/9721691

**Published:** 2022-07-07

**Authors:** Wei Miao, Honghui Zhou

**Affiliations:** ^1^School of Textile Garment and Design, Changshu Institute of Technology, Changshu 215500, China; ^2^College of Materials Science and Engineering, Northeast Forestry University, Harbin 150040, China

## Abstract

With the continuous progress of the economic era, both art and design education and local small and medium-sized enterprises are facing the crisis of survival and the pressure of competition, forcing the two to join hands to resist this crisis. The protection of the ecological environment will not only affect people's lives, but also affect the design and creation of art. This paper adopts the methods of correlation degree and correlation coefficient to construct a feasibility analysis model of mutual benefit cooperation between environment-embedded art and design education and local SMEs development based on improved grey analysis. It is to help art and design education and local small and medium-sized enterprises to continue to develop. The research results of this paper show that: (1) The accuracy of the model in this paper is on the rise as a whole, with the highest accuracy rate of 96.2%; the highest accuracy rate of the improved neural network model is 87.1%; the highest accuracy rate of the random forest algorithm is 86.3%; and the traditional model is the highest. The accuracy rate is 80.3%. (2) The recall rate of the traditional model is between 0.0816 and 0.0984; the recall rate of the random forest algorithm is between 0.726 and 0.983; the recall rate of the improved neural network is between 0.752 and 0.961; the recall rate of the model in this paper is between 0.615 and 0.815. (3) The overall static payback period is decreasing year by year, and the overall rate of return is also increasing year by year, which shows that the cooperation between art and design education and enterprises can bring higher benefits to enterprises. (4) After the cooperation between the two companies in 2016, various indicators have risen significantly. The highest net present value is 92.55 million yuan; the highest profit index is 1.98; the highest net present value rate is 35.8%, and the highest internal rate of return is 79.2%. (5) After school 2 cooperates with the enterprises, the employment rate has increased year by year, with the highest employment rate of 88.3%. In contrast, the annual employment rate of school 1, which does not cooperate with enterprises, is irregular. (6) The percentages of environmental indicators such as total emission reduction, environmental quality, and pollution control have all increased, and resource consumption has decreased by 28%; the public's satisfaction with the results of environmental protection has also reached 90%. (7) The average evaluation of each index is above 8 points, the highest score for completeness is 8.5, the highest score for feasibility is 8.9, the highest score for recognition is 9.2, and the highest score for practicality is 8.7.

## 1. Introduction

As the economy continues to develop and improve, both art and design education and local SMEs are struggling. Art and design education promotes the development of local small and medium-sized enterprises, and local small and medium-sized enterprises also provide a guarantee for art and design education, and the two promote and cooperate with each other. Human beings are both creators and shapers of the environment, but in many areas, people can see signs of pollution in large areas, and the polluted environment is incompatible with the artistic beauty. In order to protect the environment and promote environmental awareness, it is also an obligation as an art designer. This paper adopts the methods of correlation degree and correlation coefficient to construct a feasibility analysis model of mutual benefit cooperation between environment-embedded art and design education and local SMEs development based on improved grey analysis. In order to better analyze these two possibilities, achieve the ideal goal of mutual benefit. This paper has received a lot of support based on the research results so far. Grey analysis is a method of multivariate statistical analysis [1]. The concept of grey is associated with the white system and the black system [2]. Grey relational analysis can be used not only for relational analysis, but also for evaluation [3]. The grey analysis reflects the degree of correlation between the curves [4]. Grey analysis method is a method to measure the correlation between factors according to the similarity or dissimilarity of development tendency between factors [5]. Generally speaking, grey analysis can be used to analyze the degree of influence of various factors on the results [6]. Grey system theory is a system science theory developed by Professor Deng Julong [7]. The application of grey analysis includes various fields of social sciences and natural sciences [8]. Correlation is divided into absolute correlation and relative correlation [9]. Art and design education can improve people's awareness and understanding of beauty [10]. Its basic purpose is to develop balanced people [11]. Feasibility analysis is a comprehensive system analysis method that provides the basis for project decision-making [12]. Feasibility analysis is predictable, fair, reliable, and scientific [13]. Feasibility analysis is an important activity at the beginning of a project [14]. It is very important for the entire national economy [15].

## 2. Basic Knowledge

### 2.1. Grey Analysis

#### 2.1.1. Concept

Grey Analysis [16]. It is based on grey system theory to deal with complex systems in research, and uses a series of methods such as grey generation, grey correlation analysis, grey cluster analysis, and grey prediction to maximize the use of collected information. Choose a reasonable generation method. The actual samples of each clustered object are qualitatively and quantitatively analyzed by the whitening function of abstract dimension and spatial series curve fitting and GM modeling prediction.

The basic idea of grey analysis is relative ranking analysis. This is based on the similarity of the geometric shapes of the sequential curves to judge whether they are closely related. It is also a method for quantitatively describing and comparing the state of system development.

### 2.2. Grey Analysis Method

The purpose of grey analysis is to quantitatively characterize the degree of correlation between various factors, to find the main relationship of various factors in the system, to find out the important factors that affect the development of the system, and to grasp the main characteristics.

#### 2.2.1. Data Transformation

The physical meaning of each element in the system is different, or the measurement unit is different, so the dimension of the data is different. And sometimes the magnitudes of the values are very different. If the dimension and the number of digits are different, it is inconvenient, or it is difficult to obtain the correct result during the comparison process. To facilitate analysis, the raw data must be processed before comparing the elements [17].

*(1) Initial value processing*. All data of a sequence is removed by its first number, and the method of obtaining a new sequence is called initializing. The sequence shows the multiples of different time values of the original sequence compared to the first value. The sequence has a common starting point, is dimensionless, and the data in the data are all greater than 0.With original sequence

(1) $$\begin{array}{c} x^{\left(0\right)}\left(i\right)=\left\{x^{\left(0\right)}\left(1\right),x^{\left(0\right)}\left(2\right),\ldots ,x^{\left(0\right)}\left(n\right)\right\}. \end{array}$$

After initializing *x*^(0)^(*i*) to get *x*^(1)^(*i*), then

(2) $$\begin{array}{c} x^{\left(1\right)}\left(i\right)=\left\{x^{\left(0\right)}\left(1\right)/x^{\left(0\right)}\left(1\right),x^{\left(0\right)}\left(2\right)/x^{\left(0\right)}\left(1\right),\ldots ,x^{\left(0\right)}\left(n\right)/x^{\left(0\right)}\left(1\right)\right\},\\ x^{\left(1\right)}\left(i\right)=\left\{x^{\left(1\right)}\left(1\right),x^{\left(1\right)}\left(2\right),\ldots ,x^{\left(1\right)}\left(n\right)\right\}. \end{array}$$

*(2) Average processing*. The method of removing all data of a series by its average value to obtain a new series is called mean processing. This new array indicates the multiples of the values at different times in the original array relative to the mean. The method of dividing all the data in a series by the mean and obtaining a new series is called averaging. This new series shows the multiples of the values of the original array at different time points relative to the mean.

With original sequence

(3) $$\begin{array}{c} x^{\left(0\right)}\left(i\right)=\left\{x^{\left(0\right)}\left(1\right),x^{\left(0\right)}\left(2\right),\ldots ,x^{\left(0\right)}\left(n\right)\right\}. \end{array}$$

Do the mean processing on *x*^(0)^(*i*), and get *x*^(1)^(*i*) as

(4) $$\begin{array}{c} x^{\left(1\right)}\left(i\right)=\left\{x^{\left(0\right)}\left(1\right)/x^{\left(0\right)},x^{\left(0\right)}\left(2\right)/x^{\left(0\right)},\ldots ,x^{\left(0\right)}\left(n\right)/x^{\left(0\right)}\right\},\\ x^{\left(1\right)}\left(i\right)=\left\{x^{\left(1\right)}\left(1\right),x^{\left(1\right)}\left(2\right),\ldots ,x^{\left(1\right)}\left(n\right)\right\}. \end{array}$$

In

(5) $$\begin{array}{c} x^{\left(0\right)}=\frac{1}{n}\sum_{k=1}^{n}x^{\left(0\right)}\left(k\right). \end{array}$$

#### 2.2.2. Correlation Coefficient

The degree of correlation between systems or factors judges whether they are closely related according to the degree of similarity in geometry between the curves. Therefore, a measure of the degree of association between curves can be used as a measure of the degree of association [18].

Let the parent factor sequence {*x*_0_(*i*)} and the child factor sequence {*x*_*j*_(*i*)} be, respectively,

(6) $$\begin{array}{c} x_{0}\left(i\right)=\left\{x_{0}\left(1\right),x_{0}\left(2\right),\ldots ,x_{0}\left(n\right)\right\},\\ x_{j}\left(i\right)=\left\{x_{j}\left(1\right),x_{j}\left(2\right),\ldots ,x_{j}\left(n\right)\right\}, \end{array}$$

Of which *i*=1,2,…, *n*;  *j*=1,2,…, *m*. The correlation coefficient *ξ*_0*j*_(*i*) between {*x*_0_(*i*)} and {*x*_*j*_(*i*)} can be expressed by the following relation:

(7) $$\begin{array}{c} \xi_{0j}\left(i\right)=\frac{\underset{j}{\min}\underset{i}{\min}\left|x_{0}\left(i\right)-x_{j}\left(i\right)\right|+\rho \underset{j}{\max}\underset{i}{\max}\left|x_{0}\left(i\right)-x_{j}\left(i\right)\right|}{\left|x_{0}\left(i\right)-x_{j}\left(i\right)\right|+\rho \underset{j}{\max}\underset{i}{\max}\left|x_{0}\left(i\right)-x_{j}\left(i\right)\right|}. \end{array}$$

Among them, *ξ*_0*j*_(*i*) is called the correlation coefficient of *x*_0_ to *x*_*j*_ at time *i*.

Write down the minimum absolute value difference between the two levels at each moment as

(8) $$\begin{array}{c} \nabla_{\min}=\underset{j}{\min}\underset{i}{\min}\left|x_{0}\left(i\right)-x_{j}\left(i\right)\right|. \end{array}$$

The maximum absolute value difference between the two levels is recorded as

(9) $$\begin{array}{c} \nabla_{\max}=\underset{j}{\max}\underset{i}{\max}\left|x_{0}\left(i\right)-x_{j}\left(i\right)\right|. \end{array}$$

#### 2.2.3. Relevance

A measure of the magnitude of the correlation between two systems or two factors is called the degree of correlation [19]. The degree of correlation represents the relative change between factors in the system development process, that is, the relativity of the magnitude, direction, and speed of the change. A correlation between two is considered large if two relative changes during development are substantially the same. Otherwise, the correlation between the two becomes smaller.

The degree of association is denoted as *r*_0*j*_, and its expression is

(10) $$\begin{array}{c} r_{0j}=\frac{1}{N}\sum_{i=1}^{N}\xi_{0j}\left(i\right). \end{array}$$

Among them, *r*_0*j*_ represents the degree of correlation between the sub-number sequence *j* and the parent sequence 0 [20]. *N* represents the length of the sequence, that is, the number of data [21].

(1) Dun's correlation degree
  (11) $$\begin{array}{c} r\left(x_{0},x_{i}\right)=\frac{1}{n}\sum_{i=1}^{n}r\left(x_{0}\left(k\right),x_{i}\left(k\right)\right), \end{array}$$
In
  (12) $$\begin{array}{c} r\left(x_{0}\left(k\right),x_{i}\left(k\right)\right)=\frac{\underset{i}{\min}\underset{k}{\min}\left|x_{0}\left(k\right)-x_{i}\left(k\right)\right|+\rho \underset{i}{\max}\underset{k}{\min}\left|x_{0}\left(k\right)-x_{i}\left(k\right)\right|}{\left|x_{0}\left(k\right)-x_{i}\left(k\right)\right|+\rho \underset{i}{\max}\underset{k}{\min}\left|x_{0}\left(k\right)-x_{i}\left(k\right)\right|}, \end{array}$$
*ρ* is the resolution factor, and *ρ* ∈ [0,1].
(2) Grey absolute correlation degree
  (13) $$\begin{array}{c} \varepsilon_{0i}=\frac{1+\left|s_{0}\right|+\left|s_{i}\right|}{1+\left|s_{0}\right|+\left|s_{i}\right|+\left|s_{i}-s_{0}\right|}, \end{array}$$
the absolute correlation degree is the grey absolute correlation degree obtained by considering the polygonal change of the curve relative to the starting point, that is, by moving the starting point of the data series curve to the coordinate point and checking its proximity.
(3) Relative degree of correlation
Let *X*_0_ and *X*_*i*_ have the same length, and the initial value may not be equal to zero [22]. *X*_0_′ and *X*_*i*_′ are the initial value images of *X*_0_ and *X*_*i*_, respectively, then the absolute grey correlation degree of *X*_0_′ and *X*_*i*_′ is called the grey-relative correlation degree of *X*_0_ and *X*_*i*_, which is referred to as the relative correlation degree and denoted as *r*_0*i*_.
  (14) $$\begin{array}{c} r_{0i}=\frac{1+\left|s_{0}^{\prime }\right|+\left|s_{i}^{\prime }\right|}{1+\left|s_{0}^{\prime }\right|+\left|s_{i}^{\prime }\right|+\left|s_{i}^{\prime }-s_{0}^{\prime }\right|}, \end{array}$$
the relative degree of correlation is the absolute degree of grey-scale correlation of the initialized sequence calculated after initializing the original sequence. The grey-scale absolute correlation is the proximity of the absolute values of the sequence polygons, and the grey-relative correlation is the proximity of the absolute values of the sequence polygons. This formula is used to investigate the closeness of the rate of change of a series of polygons relative to the starting point. The grey relative and grey absolute relevance are calculated in the same way, so the range of applicable sequences is also the same, but the starting points of the two objects are different.
(4) Slope correlation
  (15) $$\begin{array}{c} \varepsilon_{i}=\frac{1}{n-1}\sum_{t=1}^{n-1}\xi_{i}\left(t\right). \end{array}$$

The slope correlation mainly considers the vicinity of the slope between the data series curves, so the internal slope of the data series needs to be calculated, but since the internal slope of the indicator series cannot be calculated, it is only suitable for time series.

### 2.3. Grey Analysis Model

(1) The dimensionlessization of the evaluation factor is aimed at eliminating incommensurability.
There is *m* evaluation factor *x*_1_, *x*_2_, ..., *x*_*m*_ and *n* objects participating in the evaluation, then the original data matrix *x*_*ij*_ can be obtained. Depend on
  (16) $$\begin{array}{c} P_{ij}=\frac{x_{ij}}{\sum_{j=1}^{n}x_{ij}},\;\left(j=1,2,\ldots ,n\right). \end{array}$$
The dimensionless evaluation factors can be obtained.
(2) Find the absolute difference
  (17) $$\begin{array}{c} z_{ij}=\left|p_{ij}-p_{ij\max}\right|,\;\left(i=1,2,\ldots ,m\right), \end{array}$$
and find its maximum value *z*_*j*max_′ and minimum value *z*_*j*min_′, where (*j*=1,2,…, *n*) .
(3) Find the maximum value *z*_max_^″^ and the minimum value*z*_min_^″^ of *z*_*j*max_′ and *z*_*j*min_′(*j*=1,2,…, *n*).
(4) Find the correlation coefficient.
Use the formula:
  (18) $$\begin{array}{c} \xi_{ij}=\frac{z_{\min}^{\prime \prime }+0.5z_{\max}^{\prime \prime }}{z_{ij}+0.5z_{\max}^{\prime \prime }},\;\left(i=1,2,\ldots ,m,\;j=1,2,\ldots ,n,\;\rho =0.5\right), \end{array}$$
(5) Find the correlation degree *r*_*i*_ of each factor.
  (19) $$\begin{array}{c} r_{i}=\frac{1}{n}\sum_{j=1}^{n}\xi_{ij},\;\left(i=1,2,\ldots ,m\right), \end{array}$$
when *r*_*i*_ is larger, the importance of index *x*_*i*_ in each evaluation factor is stronger, which reflects the closeness and influence of the comparison sequence and the reference sequence.
(6) Calculate the weights of each item *w*_*i*_
Use the formula:
  (20) $$\begin{array}{c} w_{i}=\frac{r_{i}}{\sum_{i=1}^{m}r_{i}}. \end{array}$$

From this, the weight of each evaluation factor can be obtained. It is shown in Figure 1.

The grey analysis model first needs to initialize the original measurement data, how to initialize the original data, then calculate the absolute difference, the two-level maximum difference and the minimum difference, calculate the maximum difference and the minimum difference, calculate the correlation coefficient, and finally calculate the correlation degree and print the association matrix.

## 3. Feasibility Analysis of Environment-Embedded Art and Design Education and Mutually Beneficial Cooperation in the Development of Local Small and Medium-Sized Enterprises

### 3.1. Environment Embedding

Environment refers to environmental protection, ecological environment pollution, etc. Embedded means firmly fixed or established. Environmental embeddedness is guided by national goals or strategic needs, in-depth art and design education process, and raising people's value expectations for education. Environment-embedded art design education is to protect the environment, protect ecological balance, and promote environmental awareness through art design. The goals and strategic needs of the country set what kind of people to cultivate for art and design education. SMEs provide talent support and market position for art and design education. Environmental embedding usually includes three levels: macro, meso, and micro.

#### 3.1.1. Macro-Level

From the macro-level environmental embedding, we will promote the high-quality reform of art and design education. Local SMEs promote economic development and guide the strategic direction of serving local economic development. Provide strong economic and technical support for art and design education. However, the current talent training in art and design education cannot meet the skills and quality requirements for the economic development of local SMEs. Art and design education needs to strengthen the implementation of quality reform to adapt to this new situation. In order to deepen the concept of cooperation with local SMEs, we will take the lead in taking measures. In the education quality reform, continuously improve the quality of personnel training and complete the reform of art and design education [23].

#### 3.1.2. Meso-Level

The environmental embedding at the mesoscopic level enhances the value expectation of artistic talents [24]. Now, the development of SMEs is very effective, the possibility of growth is high, full of vitality, with broad prospects, talent cultivation in art and design education, and the expectation and value of work are getting stronger and stronger.

#### 3.1.3. Micro-Level

From the micro-level environmental embedding, improve the adaptability of students to the employment of art and design [25]. Local small and medium-sized enterprises require educators to focus on cultivating students' artistic literacy. More than any other company in the past, they attach great importance to the talent of art and design education, and further improve the staff's requirements for comprehensive quality, knowledge, and cultural level. Through the construction of art and design education, the awareness of cooperation among art students will be continuously improved, the employability of art students will be improved, and more guarantees and opportunities will be provided for art students.

### 3.2. The Role of Environmental Protection in Art and Design Education

Art design education and environmental protection are closely linked. Art design alone and ignoring environmental protection will only damage the environment. Therefore, it is the responsibility of art design education to establish environmental protection awareness. Art design education is reflected in environmental protection, combining art design with environmental protection, beautifying people's living environment through art design, and achieving the purpose of environmental protection.

#### 3.2.1. In Interior Design

Art design should combine landscaping interior design with green environmental protection. Interior design should not only pursue beauty and comfort, but also pursue green energy conservation.

#### 3.2.2. In Daily Life

People often encounter discarded items that most people choose to throw away, and this is the act that causes our environment to be destroyed. Through art and design education, we can choose to make reasonable use of these discarded items and turn waste into treasure. This can not only reduce economic investment, but also reduce waste of resources, thereby protecting the environment.

#### 3.2.3. In the Design of Landscape Facilities

You can choose to install the energy-saving device on the locust disaster landscape facilities, which can not only bring the required energy to the landscape facilities, but also reduce the dependence on environmental resources, thus playing a role in the environmental protection.

### 3.3. The Current Situation of Art and Design Education and the Development of Local Small and Medium-Sized Enterprises

#### 3.3.1. The Development of Art and Design Education has Made Great Progress So Far

However, with the rapid development of the economy and the demand for high-level talents in modern industries, the confusion of “talented products” of art and design education and the demand for Chinese industries are becoming more and more serious. For example, in the traditional training method, the growth design talent lacks practicality and creativity, and does not meet the diverse market needs. The subject system is composed of a single repetition, without characteristics, and it is difficult to meet the needs of the multilevel market. The department of experts is too small, the boundaries of experts are too clear, and the integration of each other is insufficient. The teaching method is closed, the teaching method is not innovative, and the students cannot thoroughly practice learning.

#### 3.3.2. Development Status of Small and Medium-Sized Enterprises

Compared with large enterprises, SMEs are more innovative and dynamic. However, it is disadvantageous in terms of scale and strength, and SMEs in the development stage do not want to spend a lot of money on the design and planning of corporate image and product appearance. Products that symbolize low prices and low quality, lack of independent brands, lack of product design and development after technical level, lack of long-term corporate image and product development and design plans, etc., all limit the long-term development of enterprises.

#### 3.3.3. Analysis of the Relationship between Art and Design Education and Local SMEs

In developed countries, art and design education takes the form of a studio. Enterprises and universities cooperate to implement product research and development, design, packaging, publicity, etc., and use each other to bring benefits to each other. In recent years, many universities in our country have also adopted this method, but it has no substantial effect. Art and design education and small and medium-sized enterprises are independent, there is no complementary advantage, there is no resource sharing and mutually beneficial cooperation system. The favorable resources for artistic talents are wasted in large quantities, and small and medium-sized enterprises have been ignoring the careful development of products because of problems such as capital and thinking concepts, and the two have not entered the virtuous circle of the market economy.

### 3.4. The Practical Value of Mutually Beneficial Cooperation between Art and Design Education and the Development of Local SMEs

Facing today's market economy, art and design education and small and medium-sized enterprises will face development opportunities and fierce competition pressure. Art and design education should be helpful to local SMEs. There is a need to promote the development of art and design education. In order to have a broader development space, the two complement each other and cooperate with each other.

#### 3.4.1. Improve the Competitiveness of Enterprises and the Added Value of Products

The development of small and medium-sized enterprises is the bright spot of local economic development and the most powerful main force of local economy. Art and design education is historically important for improving the possibility of developing small and medium-sized enterprises, producing high-value-added high-end products, forming a benign corporate operation track, and creating an independent corporate brand.

#### 3.4.2. Improve Social Awareness and Brand Competitiveness

Today, education is completely introduced into the market, and design education is faced with both hot and difficult issues such as financing, registration, and employment. The training of design talents, in order to meet the needs of the market and promote the development and growth of the enterprise, needs the financial support of the enterprise. The growth of the enterprise provides an important guarantee for education, and puts forward higher educational requirements and goals.

#### 3.4.3. Improve Product Quality Standards for Design Talents and Solve Local Employment Problems

To cultivate highly innovative and practical art design talents for the society is the basic goal of art design education. SMEs have played an important role in the reform of art and design education, the establishment of the foundation of educational practice, and the transformation of educational outcomes.

#### 3.4.4. Accelerate the Transformation of Scientific Research Achievements in Art Design

Education is the main source of knowledge innovation, the driving force of the economy, and the driving force of enterprise reform. SMEs have excellent resources for capital and industrial implementation. Two double-edged swords, combining resources to complement each other, in-depth cooperation, improving their respective market adaptability and innovation vitality, effectively combining cultural, scientific research and economic interests, transforming cultural productivity into social productivity, and promoting the healthy development of local economy.

## 4. Experimental Analysis

### 4.1. Model Testing

This article conducts feasibility analysis based on the grey analysis model. This part needs to test the grey analysis model and compare the grey analysis model with the improved neural network and random forest algorithm and traditional models. The experiment selects the enterprise income after the cooperation between a university's art design and small and medium-sized enterprises as the experimental data.

Comparing the accuracy of different models on the results of cooperation between art and design education and SMEs, the results are shown in Figure 2.

As can be seen from Figure 2, the overall accuracy of the model in this paper is on the rise, but it has declined in 2018. The highest accuracy rate is 96.2% and the lowest accuracy rate is 86.7%; the overall upward trend of the improved neural network model is not obvious, and it is rising. There were two downward trends in the process, the highest accuracy rate was 87.1%, and the lowest accuracy rate was 80.7%; the overall random forest algorithm also showed an upward trend, and it rose slowly after 2017, with the highest accuracy rate of 86.3% and the lowest accuracy rate. The accuracy rate of the traditional model is the lowest, although the increase is more obvious, the highest accuracy rate is 80.3%, but the lowest accuracy rate is 70.3%. It can be seen that the grey analysis model proposed in this paper has a high accuracy.

On this basis, in order to further verify the effectiveness of the grey analysis model, the recall rate of the results of cooperation between art design education and small and medium-sized enterprises was used as an experimental indicator to test the performance of different models. The recall rate is inversely proportional to the accuracy rate. When the recall rate is low, the accuracy rate is high, which proves that the effectiveness of the model is higher. The recall rates of different models are shown in Figure 3.

As can be seen from Figure 3, the recall rate of the traditional model is between 0.0816 and 0.0984; the recall rate of the random forest algorithm is between 0.726 and 0.983; the recall rate of the improved neural network is between 0.752 and 0.961; the recall rate of this model is 0.615–0.815. It can be clearly seen from the experimental results that the recall rate of the model in this paper is smaller than that of the other three models. According to the high accuracy rate when the recall rate is low, it can be concluded that the model in this paper is more effective.

### 4.2. Feasibility Analysis

In order to better reflect the feasibility of mutual beneficial cooperation between art and design education and local small and medium-sized enterprises, this article compares the static and dynamic indicators of local small and medium-sized enterprises before and after cooperation with art and design education and the advantages of mutually beneficial cooperation. The feasibility analysis indicators of mutual benefit cooperation between art design education and local SMEs can be divided into static indicators and dynamic indicators. Static indicators are static payback period and rate of return; dynamic indicators are net present value, net present value rate, profit index, and internal rate of return.

#### 4.2.1. Static Indicators

In order to analyze whether the mutual cooperation between art and design education and local SMEs can bring better benefits to enterprises, this article compares the static indicators before and after cooperation. The experiment will make art and design education and local SMEs in 2016. Carry out mutually beneficial cooperation and calculate the value of various static indicators from 2014 to 2015. The results are shown in Table 1:

It can be seen from Figure 4 that the overall static payback period is decreasing year by year, but the static payback period is increasing before the mutual benefit cooperation between art and design education and local SMEs. The highest static payback period is 3.5 years, and it is reduced to 1.3 years. The overall rate of return is also increasing year by year, but the rate of return is decreasing before the mutual cooperation between art and design education and local small and medium-sized enterprises. The lowest rate of return is 61.4% and the highest rate of return is 87.8%. It shows that the cooperation between art and design education and enterprises can bring higher benefits to enterprises.

#### 4.2.2. Dynamic Indicators

In order to analyze whether the mutual benefit cooperation between art and design education and local small and medium-sized enterprises can bring better benefits to enterprises, this article will also compare the dynamic indicators before and after cooperation. Enterprises conduct mutually beneficial cooperation and calculate the value of various dynamic indicators from 2014 to 2015. The results are shown in Table 2:

As can be seen from Figure 5, various dynamic indicators generally show an upward trend, and the indicators are still decreasing before the cooperation between art and design education and enterprises. After the cooperation between the two parties in 2016, various indicators have risen significantly. The highest net present value is 92.55 million yuan; the highest profit index is 1.98, and the project is feasible only when the profit index is greater than 1 or equal to 1, indicating that the feasibility is fully reflected when the two cooperate; the highest net present value is 35.8%, the highest internal rate of return is 79.2%. Various dynamic indicators show that the mutual beneficial cooperation between art and design education and local small and medium-sized enterprises is feasible, and it can also bring greater benefits to small and medium-sized enterprises, and the income is increasing year by year.

### 4.3. Analysis of the Employment Situation of Art and Design Students

This article analyzes the considerable benefits that reciprocal cooperation brings to companies, as well as the benefits for art and design education students. The experiment also adopts the comparison method, selecting two colleges and universities with art and design education majors, school 1 does not cooperate with enterprises, and school 2 cooperates with enterprises, and compares the employment rate of students after graduation from 2014 to 2020 in the two colleges and universities. The result is shown in Figure 6:

It can be seen from Figure 6 that after School 2 cooperates with enterprises, the employment rate has increased year by year. Although there was a slight decline in 2016, it has not declined since 2016, with the highest employment rate of 88.3%. On the other hand, the annual employment rate of schools 1 that do not cooperate with enterprises is irregular, sometimes rising and falling, which is relatively unstable. The highest employment rate was 76.3%, which was 12% lower than the highest employment rate in School 2. It shows that schools that cooperate with enterprises have higher employment rates and provide more job opportunities for students.

### 4.4. Comparison of Environmental Protection

This article also compares the environmental protection indicators before and after the cooperation between art and design education and local small and medium-sized enterprises. The comparison indicators are total emission reduction, resource consumption, environmental quality, pollution control, and public satisfaction with environmental protection. The results are shown in Figure 7.

As can be seen from Figure 7, the percentages of environmental indicators such as total emission reduction, environmental quality, and pollution control are all increasing, and the increase rate is large; resource consumption is decreasing by 28%. Satisfaction also reached 90%. It shows that the cooperation between the two has played an obvious role in environmental protection and should be vigorously promoted.

### 4.5. Feasibility Evaluation

The environment embedded art design education based on improved grey analysis and the mutually beneficial cooperation with local small and medium-sized enterprises still need to be evaluated by people from all walks of life. In the experiment, experts in different fields, as well as students and business entities were invited to evaluate the various indicators of the cooperation. If the average value of each indicator is above 8 points, it means that the cooperation is feasible. The result is shown in Figure 8:

As can be seen from Figure 8, experts, students, and business entities have high evaluations of the reciprocal cooperation proposed in this paper. The average evaluation of each index is above 8 points. The highest score for completeness is 8.5, and the highest score for feasibility is 8.9, the highest score for recognition is 9.2, and the highest score for practicality is 8.7. It shows that art and design education is feasible for local SMEs to develop mutually beneficial cooperation.

## 5. Conclusion

With the increasing number of college graduates year by year, it is also a big problem for college students to find jobs, and in the face of market competition, small and medium-sized enterprises do not have an advantage. Based on this phenomenon, this article proposes that art and design education and local small and medium-sized enterprises develop mutually beneficial cooperation, so that art and design education can serve small and medium-sized enterprises, and small and medium-sized enterprises can promote the development of art and design education, and play the ultimate goal of environmental protection. This article adopts the method of correlation degree and correlation coefficient to construct a feasibility analysis model based on improved grey analysis of environment-embedded art and design education and the development of mutual benefit cooperation between local SMEs. In order to make art and design education and local SMEs develop together in a better direction.

The findings of the article show that:

1. The accuracy rate of the model in this paper is on the rise as a whole, with the highest accuracy rate of 96.2% and the lowest accuracy rate of 86.7%; the overall upward trend of the improved neural network model is not obvious, and the highest accuracy rate is 87.1%. In the upward trend, the highest accuracy rate is 86.3%; while the traditional model has the lowest accuracy rate, the highest accuracy rate is 80.3%. It can be seen that the grey analysis model proposed in this paper has a high accuracy.
2. The recall rate of the traditional model is between 0.0816 and 0.0984; the recall rate of the random forest algorithm is between 0.726 and 0.983; the recall rate of the improved neural network is between 0.752 and 0.961; the recall rate of the model in this paper is between 0.615 and 0.815. From the experimental results, it is obvious that the model in this paper is more effective.
3. The overall static payback period shows a decreasing trend year by year, the highest static payback period is 3.5 years, and the decrease is 1.3 years. The overall rate of return is also increasing year by year, the lowest rate of return is 61.4%, and the highest rate of return is 87.8%. It shows that the cooperation between art and design education and enterprises can bring higher benefits to enterprises.
4. The overall dynamic indicators showed an upward trend. After the cooperation between the two parties in 2016, the indicators increased significantly. The highest net present value is 92.55 million yuan; the highest profit index is 1.98; the highest net present value rate is 35.8%, and the highest internal rate of return is 79.2%. Various dynamic indicators show that the mutual beneficial cooperation between art and design education and local small and medium-sized enterprises is feasible, and it can also bring greater benefits to small and medium-sized enterprises, and the income is increasing year by year.
5. After school 2 cooperates with enterprises, the employment rate has increased year by year, with the highest employment rate of 88.3%. On the other hand, the annual employment rate of schools 1 that do not cooperate with enterprises is irregular, sometimes rising and falling, which is relatively unstable. It shows that the schools that cooperate with enterprises have higher employment rates and provide more job opportunities for students.
6. The percentages of environmental indicators such as total emission reduction, environmental quality, and pollution control are all on the rise, and the rate of increase is large; resource consumption is decreasing by 28%; the public's satisfaction with the results of environmental protection has also reached 90%. It shows that the cooperation between the two has played an obvious role in environmental protection and should be vigorously promoted.
7. The average evaluation of each indicator by experts, students, and business entities is above 8, the highest score for completeness is 8.5, the highest score for feasibility is 8.9, the highest score for recognition is 9.2, and the highest score for practicality is 8.5. The highest score was 8.7. It shows that art and design education is feasible for local SMEs to develop mutually beneficial cooperation.

In order to promote mutually beneficial cooperation between art and design education and local small and medium-sized enterprises, it is necessary to establish a discipline system of art and design education with local economic characteristics; formulate a talent training model for art and design education with local economic characteristics; strengthen school-enterprise cooperation;, realize the personalized training of talents; actively promote the achievements of art and design scientific research to local small and medium-sized enterprises, and realize the transformation of knowledge into economic wealth. Although the experimental results in this paper have obvious advantages, they still have certain limitations. This model is limited to art and design education, and it is not obvious in other majors. It is hoped that further research can be carried out on the scope of application in the following research to increase the universality of the model.

## Figures and Tables

**Figure 1:** Grey analysis model.

**Figure 2:** Accuracy comparison.

**Figure 3:** Comparison of recall rates.

**Figure 4:** 2014–2020 static indicators.

**Figure 5:** Dynamic indicators from 2014 to 2020.

**Figure 6:** Analysis of student employment situation.

**Figure 7:** Comparison of environmental protection.

**Figure 8:** Feasibility evaluation.

**Table 1:** 2014–2020 static indicators.

Index	2014	2015	2016	2017	2018	2019	2020
Static payback period	3.4	3.5	2.8	2.5	2.2	1.6	1.3
Rate of return	63.8%	61.4%	70.3%	72.6%	75.8%	83.4%	87.8%

**Table 2:** Dynamic indicators from 2014 to 2020.

Index	2014	2015	2016	2017	2018	2019	2020
Net present value (ten thousand yuan)	6757	5938	7982	8326	8746	8927	9255
Net present value rate	16.7%	14.4%	21.4%	26.3%	29.1%	32.4%	35.8%
Profitability index	0.87	0.63	1.72	1.76	1.63	1.98	1.98
Internal rate of return	58.2%	54.8%	61.7%	62.8%	74.3%	77.8%	79.2%

## Data Availability

The experimental data used to support the findings of this study are available from the corresponding author upon request.
